RETRACTED

# Identifying a 6-Gene Prognostic Signature for Lung Adenocarcinoma Based on Copy Number Variation and Gene Expression Data

**DOI:** 10.1155/2022/6962163

**Published:** 2022-09-28

**Authors:** Yisheng Huang, Liling Qiu, Xiaoye Liang, Jing Zhao, Haoting Chen, Zhiqiang Luo, Wanzhen Li, Xiaohua Lin, Jingjie Jin, Jian Huang, Gong Zhang

**Affiliations:** ^1^Postdoctoral Innovation Center of Zhongshan Chenxinghai Hospital, Jinan University, Guangzhou, China; ^2^Department of Oncology, Maoming People's Hospital, Maoming City, China; ^3^Key Laboratory of Functional Protein Research of Guangdong Higher Education Institutes, Institute of Life and Health Engineering, College of Life Science and Technology, Jinan University, Guangzhou, China; ^4^Department of Endocrinology, Zhongshan Hospital of Sun Yat-Sen University, Zhongshan City People's Hospital, Zhongshan City, China; ^5^Translational Medicine Center, Key Laboratory of Molecular Target and Clinical Pharmacology, School of Pharmaceutical Sciences, The Second Affiliated Hospital of Guangzhou Medical University, Guangzhou, China; ^6^Department of Thoracic Surgery, Maoming People's Hospital, Maoming City, China

## Abstract

The occurrence of lung adenocarcinoma (LUAD) is a complicated process, involving the genetic and epigenetic changes of proto-oncogenes and oncogenes. The objective of this study was to establish new predictive signatures of lung adenocarcinoma based on copy number variations (CNVs) and gene expression data. Next-generation sequencing was implemented to obtain gene expression and CNV information. According to univariate, multivariate survival Cox regression analysis, and LASSO analysis, the expression profiles of lung adenocarcinoma patients were screened and a risk score formula was established and experimentally validated in a local cohort. The model was evaluated by three independent cohorts (TCGA-LUAD, GSE31210, and GSE30219), and then validated by clinical samples from LUAD patients. A total of 844 CNV-related differentially expressed genes (CNV-related DEGs) were identified. These genes are significantly associated with the imbalance of various oxidative stress pathways. A CNV-associated-six gene signature was dramatically linked to overall survival in lung adenocarcinoma samples from both training and validation groups. Functional enrichment analysis further revealed involvement of genes in p53 signaling pathway and cell cycle as well as the mismatch repair pathway. Risk score is an independent marker considering clinical parameters and had better prediction in clinical subpopulation. The same signature also classified tumor tissues of clinical patients with CNV detected from their corresponding nontumorous tissues with an accuracy of 0.92. In conclusion, we identified a new class of 6 CNV-related gene markers that may act as efficient prognostic predictors of lung adenocarcinoma, thus contributing to individualized treatment decisions in patients.

RETRACTED

## 1. Introduction

Lung cancer is the leading cause of cancer-related deaths worldwide [1]. Non-small cell lung cancer (NSCLC) counts for over 80% of total lung carcinomas, and lung adenocarcinoma is the predominant form of NSCLC. There are many patients diagnosed as distant metastases in their first consultation. For those minor early metastatic lesions cannot be detected in a proper imaging examination, a proper treatment is also difficult. [2] Although the overall survival rates of lung cancer patients are increasing with the improving technology and accessibility of therapies, the 5-year postdiagnosis survival rates were still below 20% [3–7]. The organ collapses and malfunctions connected with remote metastases were a major cause of oncology-related mortality [8]. Therefore, the technology could achieve an early-stage diagnosis, also in the treatments, the progression of precancerous lesions to invasive cancer could be prevented, thus improving the prognosis of patients.

In some long-term stage of tumorigenesis, the accumulation of multiple genetic variants promotes the occurrence and progression of tumors [9]. Copy number variation (CNV) is an important factor of gene expression changes. Recent research shows that the integrated analysis of comparative genome hybrid chip and gene expression profiling chip data provides a new perspective and revealed some molecular mechanism underlying gene expression changes [10–13]. Copy number plays a key role in cancer research in which CNV variations accounts approximately 12% of gene expression changes in breast cancer [14], and mRNA expression levels consistent with CNV regions were also observed in several genes in the lung cancer CNV regions [15, 16]. For example, studies based on targeted sequencing of protein-coding genes and single nucleotide polymorphism (SNP) arrays or whole genome/exome sequencing have found somatic mutations, local amplification, or copy number changes of many oncogenes and oncogenes (e.g., RIT1 and MGA) in LUAD patients [17, 18]. Fluorescence in situ hybridization (FISH) analysis revealed that the increased c-MYC copy number was correlated with adverse prognosis in 19% of LUAD patients [19]. Epidermal growth factor receptor (EGFR) gene amplification is also associated to LUAD tumorigenesis [20]. In addition, gene copy number has been shown to be helpful in predicting survival in lung cancer patients [21, 22]. For instance, the over expression and amplification of EGFR, and the low expression and deletion of the dual-specific phosphate 4 (DUSP4) [23], There is a strong correlation between those two factors, each of which can serve as a valid prognostic biomarker for lung cancer [16].

RETRACTED

Numerous studies have seen gene expression levels or epigenetic modification as cancer markers [24, 25]. However, due to the complex nature of LUAD, single gene expression signature is not informative on the prognosis of LUAD. Indeed, no such single-gene biomarker has been used in clinical practice for the prognosis of LUAD. Some studies tried to propose multigene signatures based on their expression. However, the relatively low AUC (area under curve) values prevented them from wide application. The altered gene expression is obviously important, but the way they dysregulated such as SNV and CNV methylation is more critical for understanding the mechanism of tumorigenesis. Therefore, the prognostic value of CNV-related DEGs in LUAD should be worth investigation for the prognosis of LUAD.

In this study, we carried out analysis of DEGs and CNVs simultaneously in TCGA lung adenocarcinoma samples. A total of 844 CNV-related genes that were variably expressed in tumor tissues and normal tissues were characterized. In which six CNV-associated gene signatures were identified in an order. The ability of six CNV-associated genetic markers to be prognostic was validated in two independent local cohorts, demonstrating their clinical significance as promising biomarkers for lung adenocarcinoma. Our data may provide additional evidence for prognostic biomarkers and therapeutic targets for LUAD.

## 2. Materials and Methods

### 2.1. Data Acquisition

We gained the latest expression profile, CNV data and clinical characteristics from the Cancer Genome Atlas (TCGA) [26]. A total of 556 samples (500 tumors and 56 normal tissues) were enrolled in this study. We also downloaded the fragments per kilobase of exon model per million reads mapped (FPKM) data of LUAD from the transcriptome RNA-Sequence data in GEO database [27], incorporating 226 LUAD samples in GSE31210 dataset and 83 LUAD samples in GSE30219 dataset.

For TCGA-LUAD, samples without clinical follow-up information, survival time samples, and status samples were removed. Genes with FPKM <1 in more than half of the samples were removed. Tumor samples and normal tissue samples (Primary Solid Tumor and Solid Tissue Normal) were retained.

For GEO data, the criteria for enrollment of publicly available LUAD patient's data were as follows: samples without clinical follow-up information, survival time, and survival status were removed. The probes correspond to multiple genes were removed. Expressions with multiple gene symbols taken a median value. The clinical statistical information of the samples is shown in Table 1. The workflow of this study is presented in Figure 1.

RETRACTED

### 2.2. Tumor-Specific CNV Identification

Bedtools [28] were used to match chromosome segments in the CNV segment file to genes, and the gene segment file of the sample was obtained. Only the segment mean of somatic cell CNV with absolute value greater than 0.2 was kept for further analysis. Differential CNV fragments were identified by Chi-square test (FDR < 0.05).

### 2.3. Differentially Expressed Genes and Functional Enrichment Analysis

Limma package [29] was used to calculated the differentially expressed genes (DEGs) between tumor samples and normal samples, with thresholds of FDR < 0.01 and |log2FC| > 1. The R software package clusterProfiler [30] was used for KEGG pathway and GO function enrichment analysis, and FDR < 0.05 was selected as the significance threshold to obtain a significant pathway. In addition, we used the ssGSEA method of R software package GSVA [31] to evaluate the GO term enrichment score of each patient in the TCGA data set to obtain the oxidative stress pathway score.

### 2.4. Definition of Local Patient Cohort

The 500 samples in the TCGA dataset were divided into training sets and validation sets. To avoid random allocation bias influencing the stability of the follow-up modeling, all samples were reinserted into the randomizer group for 100 times. Grouping was conducted in accordance with the proportion of training set: validation set = 7 : 3. The most appropriate training and validation sets were selected based on the following criteria: (1) the two groups were similar in age distribution, sex, follow-up time, and proportion of patient deaths; (2) after clustering the gene expression profiles of the two randomly grouped data sets, the number of samples of dichotomy was similar. The final sample information of training and validation set obtained TCGA data are shown in Table 2. The clinical information between the training set and the test set samples is checked by Chi-square test.

### 2.5. COX Risk Analysis for Univariate Survival

A univariate Cox proportional hazard regression model was conducted for each DEGs (844 genes) using the R package survival coxph function in training dataset with *p* < 0.01.

### 2.6. Construction of the Prognostic Gene Signature

Based on the genes obtained from the univariate Cox analysis, genes were further compressed by LASSO Cox regression using the R package glmnet [32] so as to minimize the number of genes in the risk model. In addition, stepwise regression utilized the AIC red pool information criterion, which takes into consideration the statistical fit of the model and the number of fitted parameters. The stepAIC method [33] in the MASS package starts with the highest complexity model and sequentially removes one variable to reduce the AIC. Combined with prognosis-related gene expression, we established an independent prognostic model. The formula was as follows:

(1) $$\begin{array}{c} \text{Risk score}=\text{coef}\left(\text{gene i}\right)*\exp\left(\text{gene i}\right) \end{array}$$

Coef represents the coefficients and exp represents the expression levels of prognostic genes.

RETRACTED

### 2.7. Assessment of the Risk Score in TCGA Cohort and GEO Dataset

In accordance with our prognostic model, each patient in the TCGA cohort, the GSE31210 dataset, and GSE30219 dataset was allocated a risk score. In each cohort, we used the median risk score as a cutoff to classify lung adenocarcinoma patients into high-risk and low-risk groups, respectively. Survival curves were drawn by Kaplan–Meier (KM) method and log-rank tests were employed to evaluate the survival differences between the high-risk and low-risk groups. The receiver operating characteristic curve (ROC) was established by using the “timeROC” package [34], and the area under the curve (AUC) was measured to investigate the sensitivity and specificity of the model. In addition, “rms” package (http://CRAN.R-project.org/package=rms) was used to build the prognostic nomogram based on the Cox proportional hazards regression model, which was undertaken to visually reflect the relevance of individual predictors to survival in lung cancer cases. C index and calibration curves were applied to analyze the performance of the prognostic line graph.

To further assess whether our model could be used as an independent prognostic factor, age, sex, stage, T, M, and N were included as independent variables. Univariate Cox regression analyses and multivariate Cox regression analyses were used to analyze the changes of survival outcomes.

### 2.8. Clinical Validation

Twenty-two samples were enrolled in this study. There were 2 normal samples and 20 paired tumor and adjacent nontumorous tissue samples of LUAD patients collected from The Maoming People's Hospital, China. All patients underwent primary tumors resection between 2020 and 2021. None of the patients had preoperative chemotherapy or preoperative radiotherapy. Tumor staging was determined according to AJCC TNM system. All tumor information was histologically classified based on World Health Organization criteria. Pathologic, clinical, and follow-up patient information was obtained from hospital medical records. The clinical information of 20 LUAD patients is listed in Table 3.

RETRACTED

### 2.9. Experiment Summary

Manufacturer protocols are used for tissues total RNA extraction (Trizol reagent, Thermo Fisher Scientific, USA), DNA extraction (Monarch DNA purification Kits, NEB, USA), and NGS library construction (VAHTS Universal DNA Library Prep Kit for MGI/VAHTS RNA Library Prep Kit for Illumina, Vazyme, Nanjing, China). The final DNA library was sequenced at 2 × 100 paired-end mode on MGISEQ-2000 sequencer (MGI, China), RNA library was sequenced at 2 × 150 paired-end mode on NovaSeq sequencing system (Illumina, USA). The sequencing data was uploaded to the Gene Express Omnibus (GEO) database under the accession GSE197346.

### 2.10. NGS Data Analysis

Adapters were trimmed from the reads by Cutadapt, and the reads shorter than 17 nt, and low-quality sequence were discarded. The quantity of gene expression was calculated by the RPKM method (reads per kilobase per million reads), The mRNA reads were mapped to the RefSeq mRNA reference using FANSe3 algorithm FANSe3 algorithm [35] (-E5% --indel -S14). The gene expression level was quantified using RPKM method (reads per kilobase per million reads) [36]. The differential gene expression was analyzed using edgeR [37]. The genome sequencing reads were mapped to human hg19 genome from UCSC using FANSe3. All these NGS data analyses was performed in the Chi-Cloud NGS Analysis Platform (Chi-Biotech Co. Ltd., Shenzhen, China, ver.CHI.Client_V01R04C08).

## 3. Results

### 3.1. Landscape of CNV-Related DEGs in LUAD Cohort

It is known that CNV can cause the gene expression changes. However, the prognostic value of CNV-related DEGs in LUAD has not been elucidated yet. The CNV and gene expression data of LUAD patients were downloaded from the TCGA and GEO datasets. Differential CNV fragments were identified by Chi-square test (FDR < 0.05), and 7152 CNV-related genes were finally identified. Limma package was used to calculate the DEGs between tumor samples and normal samples, and 2324 DEGs were obtained according to the gene expression data (Figure 2(a)). The intersection of CNVs and DEGs was analyzed and finally 844 genes were found from both CNVs and DEGs (Figure 2(b)). These genes are mainly enriched in biological processes such as microglial cell activation, cell substrate adhesion, leucocyte activation involved in inflammatory response (Figure 2(c)), and they are also enriched in a variety of KEGG pathways, such as fructose and mannose metabolism and protein digestion and absorption (Figure 2(d)), which are closely related to tumors. It is worth mentioning that a large number of disorders of biological processes related to oxidative stress were also observed in cancer and adjacent samples, such as the activation of INTRINSIC_APOPTOTIC_SIGNALING_PATHWAY_IN_RESPONSE_TO_OXIDATIVE_STRESS pathway and the inhibition of REGULATION_OF_RESPONSE_TO_OXIDATIVE_STRESS pathway in tumor samples (Figure 2(e)). These results show that oxidative stress disorder plays an important role in lung cancer. Comparing the correlation between the expression of these 844 genes and 14 biological processes of oxidative stress, it can be observed that 838 (99.3%) genes are significantly correlated with at least one oxidative stress pathway, and the expression of most genes is significantly correlated with most biological processes of oxidative stress (Figure 2(f)).

RETRACTED

### 3.2. Determining Potential Prognostic Signature from TCGA-LUAD Cohort

The TCGA-LUAD cases (*n* = 500) were randomly divided into training and validation groups (Table 2), and there were no remarkable differences in PFS, age, pathological stage, and gender between the two groups except for the T Stage proportion (*p* < 0.001). In the training set data, by subjecting the expression profiles of 844 genes to univariate Cox proportional risk regression analysis, we identified 33 genes strongly associated (*p* < 0.01) with patient prognosis. In order to minimize the risk of overfitting, the Least Absolute Shrinkage and Selection Operator (LASSO) analysis was then performed. Lambda is the regularization parameter to control the complexity for LASSO, the greater lambda results in less variables for a multivariables linear model. As lambda gradually increases, the coefficient traces of the independent variables tend to be zero (Figure 3(a)). We used 5-fold cross-validation to construct the model and analyze the confidence interval under each lambda. At lambda =0.0296, the model achieved optimal (minimum of the partial likelihood deviation, Figure 3(b)), there still 12 genes be selected as the next objective genes.

Then stepAIC method was performed to further optimize the model and finally six candidate CNV-related DEGs were determined, including CBFA2T3, EFNB2, GOLM1, HMMR, POSTN, and TPSB2.

### 3.3. Construction and Validation of the CNV-Related DEGs Prognostic Model

In order to investigate whether the six gene signatures could exactly predict the outcome of patients with LUAD, a prognostic risk scoring model was developed based on the expression of the six genes signature as follows:

Risk score = (0.19∗EFNB2) + (0.148∗GOLM1) + (0.125∗HMMR) + (0.091∗POSTN) − (0.111∗TPSB2) − (0.189∗CBFA2T3).

The risk score of each patient in the TCGA cohorts were calculated, and patients were divided into a high-risk group (*n* = 168) and a low-risk group (*n* = 182) based on median risk score. The risk score, survival status, and gene expression heat map of these prognostic CNV-related DEGs signature (CRDS) are presented in Figure 3(c). Time-dependent ROC indicated that the AUC for 1, 3, and 5 years were 0.71, 0.69, and 0.61, respectively (Figure 3(d)). Kaplan–Meier curves showed that patients in the high-risk group had a significantly shorter overall survival (OS) than those in the low-risk group (Figure 3(e)).

RETRACTED

### 3.4. The Six Gene Signature Was Robust among LUAD and GEO Cohort

To verify the stability and the robustness of this CNV-related-six gene signature risk model, more patients from the TCGA-LUAD cohort were included to test the predictive value. We used the same model and the same coefficients in the TCGA validation set and the full dataset as in the training set and calculated the risk score for each sample separately based on the expression level of the sample.

In TCGA test cohort (*n* = 150) and entire TCGA cohort (*n* = 500), a higher overall prognosis rate was both noted for LUAD patients with low-risk scores and for those with high-risk scores. Tumor tissues from patients with high-risk scores tended to express high levels of risk mRNAs (POSTN, EFNB2, GOLM1, and HMMR), whereas tumor tissues from patients with low-risk scores tended to express high levels of protective mRNAs (TPSB2 and CBFA2T3) (Figure S1A, D). Time dependent ROC indicated that the AUC for 1, 3, and 5 years were 0.70-0.65, 0.66-0.67, and 0.66-0.83, respectively (Figure S1B, E). Kaplan–Meier curves indicated that patients in the high-risk group had a significantly shorter overall survival than those in the low-risk group (Figure S1C, F).

To further validate the robustness of the prognostic model, the same model and the same coefficients as the training set are used in the external validation sets GSE31210 and GSE30219. We also calculated the risk score for each sample separately according to the expression level of the sample. The risk score, survival status, and gene expression heat map of these prognostic genes were shown in Figure S2A, D. Time dependent ROC indicated that the AUC for 1, 3, and 5 years were also higher (Figure S2B, E). Kaplan–Meier curves demonstrated that patients in the high-risk group had a significantly shorter overall survival than those in the low-risk group in the external validation set (Figure S2C, F), which were similar to those observed in the training series.

### 3.5. Distribution of Clinical and Molecular Features among Subtypes

We evaluated the distribution of different clinical characteristics (age, gender, TNM stage, recurrence, and tumor stage) in the high- and low-risk groups, which was defined above. The results showed that high-risk pathological stages such as recurrence proportion sample, T2-4, N1-3, Stage II, III, and IV were more prevalent in the high-risk group, and that females were also more prevalent in the high-risk group (Figure S3A-G), suggesting that our model has potential for clinical application. However, we did not find the effect of M stage and age (Figure S3D, F) on the risk score.

RETRACTED

In next steps, we compared the distribution of the 10 genes with the highest mutation frequencies in the high- and low-risk groups in the TCGA dataset, and we found that TP53, TNN, MUC16, CSMD3, RYR2, LRP1B, USH2A, ZFHX4, KRAS, and XIRP2 had higher mutation frequencies in the high-risk groups than in the low-risk groups (Figure S4A, B), consistent with previous studies [38]. The mutation frequencies of all the ten genes in the high-risk groups appear a little higher than the low-risk groups.

The R software package ESTIMATE was used to calculate the immune scores for each sample separately, and showed the ImmuneScore of the low-risk group was significantly higher (*p* = 6.9E − 07) than the ImmuneScore of the high-risk group in the TCGA dataset. (Figure S4C).

### 3.6. Survival Prediction by the Prognostic Model Is Independent of Clinical Features

We found our six-gene prognostic model was still a good predictor of different clinical features (Figure S5A-P). Significant differences in T Stage, N Stage, Stage, Gender, and Smoking (*p* < 0.05) were observed by comparing the distribution of risk score between clinical feature subgroups. The risk score is higher at T Stage, N Stage, and Stage stage. In the gender grouping, risk score of Male was significantly higher than that of Female (Figure S6A-G).

Multivariate Cox regression analysis was used to assess whether six-gene signature was an independent predictor of survival in patients with lung adenocarcinoma. Univariate Cox regression analysis found that risk score, T, N Stage, and radiation-therapy were significantly correlated with survival (Figure S7A). However, after the corresponding multivariate Cox regression analysis, it showed that risktype (*p* < 1e − 5) and radiation therapy (*p* < 0.005) were still significantly correlated with prognosis (Figure S7B). As indicated above, our model has independent predictive performance in clinical application value.

### 3.7. Construction of the Nomogram

The nomogram uses the length of the line to indicate the degree of influence of difference variables on the outcome and the influence of different values of variables to predict the outcome. Based on the multivariate Cox analysis, two clinical features including radiation therapy and risk score were integrated to construct the nomogram model to evaluate their independent prognostic significance in LUAD. The nomogram suggests that risk types have the greatest influence on survival rate prediction, indicating that the risk model based on CNV-related prognostic genes can better predict prognosis (Figure 4(a)). In addition, we corrected the performance of 1, 3, and 5 years of nomogram data for visual nomograms (Figure 4(b)). DCA plots show that the prognostic model was more predictive (Figure 4(c)).

RETRACTED

### 3.8. Clinical Validation

To further validate the clinical significance of the 6-gene signature, the genomic CNV and transcriptome data of paired tumor and adjacent nontumorous tissue samples from 20 LUAD patients were performed and analyzed. To clearly examine the influence of CNVs for the CRDS, paired samples were divided to two subgroups (CNV group and Non-CNV group) by whether the tumor tissue have been detected in at least one CNV of six prognostic genes. The results showed that 55% (11/20) tumor tissues identified at least one CNV of the six prognostic genes, and those samples with its paired adjacent normal tissues were classified to CNV group, the other tumor tissues (9/20) and its paired adjacent normal tissues were classified as Non-CNV group. The medians of mRNA expression of HMMR, GOLM1, and POSTN were slightly increased, whereas TPSB2, CBFA2T3, and EFNB2 decreased in tumor tissues than in adjacent normal tissues in CNV group, although not all genes were statistically significant (Figure 5). Furthermore, comparing to Non-CNV group in Figure S8, the expressions of six genes in tumor tissues (CNV group) were higher than those genes in tumor tissues (Non-CNV group).

Significant differences were observed by comparing the distribution of risk score between adjacent nontumorous and tumor tissues groups (*p* < 0.01, Figure 6(a)), regardless of CNV in samples. And the ROC can still clearly distinguish the tumor tissues from adjacent nontumorous tissues (AUC = 0.748), confirming the robustness of the model (Figure 6(b)). Next, we divided the samples to two groups as mentioned above, the tumor tissues in CNV group have a much higher risk score than other three types of samples, also significantly higher than the tumor tissues in Non-CNV group (Figure 6(c)). Based on this result, the Figure 6(d) shows that the tumor tissues in the CNVs group can distinguish themselves from adjacent nontumorous tissues more clearly (AUC = 0.92) than those tumor samples in the Non-CNV group (AUC = 0.56). The results suggest that the risk score of the model is a crucial factor to affect the prognosis superior to other clinical risk factors, and our model is a good criterion to stratify patients in terms of prognosis.

RETRACTED

## 4. Discussion

In current studies, we collected 556 CNV-related data and mRNA expression matrixes of LUAD patients (TCGA-LUAD, GEO). In TCGA cohort, 844 CNV-related DEGs were identified between normal and tumor tissues. After screened by univariate Cox regression analysis and LASSO regression analysis, six CNV-related DEGs (*CBFA2T3*, *EFNB2*, *GOLM1*, *HMMR*, *POSTN*, and *TPSB2*) were applied in constructing a novel CNV-related DEGs signature (CRDS). Survival analysis illustrated that all of those six genes were highly related to the OS of LUAD. Of the six genes, many of these genes (*HMMR*, *EFNB2*, *GOLM1*, *CBFA2T3*, and *POSTN*) were associated with diverse human cancers, containing lung adenocarcinoma [39–43]. However, *TPSB2* has not yet been studied in association with any cancer. Identifiable genes such as *HMMR*, *EFNB2*, *GOLM1*, and *POSTN* are differentially expressed in lung adenocarcinoma lesions or are associated with patient prognosis. *HMMR* was highly expressed in LUAD tissues and cells, and HMMR knockdown suppressed cell proliferation, migration, and invasion and strengthened cell apoptosis in LUAD [44]. Xia Yang et al. reported that ephrin B2 (*EFNB2*) was confirmed to be differentially expressed in LUAD vs. normal controls at the mRNA and protein level [45]. Liu et al. showed that higher *GOLM1* expression individually determined adverse outcome and recurrence-free survival in LUAD [46]. Expression of *POSTN* in cancer-associated fibroblasts was significantly higher in NSCLC and in the adenocarcinoma and squamous cell carcinoma subtypes [47]. Interestingly, *CBFA2T3* gene is prognostic in LUAD [43], while *TPSB2* has not been studied in lung adenocarcinoma as far as we know. More investigations were necessary to discover the biological functions of these genes. The involvement in the prognostic characteristics of six genes is the first study to report their expression is associated with outcome in patients with lung adenocarcinoma. CNV values were not included in the formula, because the CNV rarely correlates the gene expression at a genome-wide scale [48]. We used CNV of these 6 genes as an indicator of genome instability. CNV-containing patients are more significantly prognosed by the 6-gene signature.

Therefore, we systematically recognized mRNA-based prognostic biomarkers by combining gene expression and copy number alterations in lung adenocarcinoma. We reported the expression characteristics of six CNV-related DEGs signature from an analysis of gene expression profile in 350 lung adenocarcinoma patients and verified the gene expression data in several independent external cohorts to accurately predict patient survival. Since the model is in combination with other clinical signs based on the overall survival of patients with stage I-IV, we consider this as a more logical and reliable prognostic gene expression feature for lung adenocarcinoma patients. Clinical validation confirmed the results and found cellular CNVs play an important role in tumorigenesis and development and affect the tumor prognosis. Although the model was constructed using the omics data from public database, we could also validate it using local patients and reach AUC = 0.92, demonstrating its efficacy and robustness.

RETRACTED

## 5. Conclusions

In summary, our study reports a robust and efficient risk profile of six genes (*CBFA2T3*, *EFNB2*, *GOLM1*, *HMMR*, *POSTN*, and *TPSB2*) associated with CNV that assist in predicting survival outcome and metastasis in LUAD patients for the first time. This discovery will help future investigators to identify new treatments for LUAD and provide additional genetic targets for the treatment of LUAD patients.

## Figures and Tables

**Figure 1:** The workflow of this study.

**Figure 2:** Identification and functional analysis of differentially expressed genes. (a) Volcano plot of differentially grouped genes between Tumor and Normal. (b) Venn diagram of CNV and differentially expressed genes. (c) The top 10 most significantly enriched biological processes enriched by differential genes. (d) The top 10 KEGG pathways enriched by differential genes. (e) Differential distribution of enrichment scores of 14 oxidative stress-related pathways in cancer and adjacent samples. (f) Number distribution of oxidative stress-related pathways significantly related to different genes.

**Figure 3:** Prognostic model construction. (a) The trajectory of each independent variable, the log of lambda on the horizontal axis and the coefficient on the vertical axis. (b) The confidence interval under each lambda. (c) Risk score, survival time and survival status and expression of 6-gene signature in the TCGA training set; (d) ROC curve and AUC of 6-gene signature in the TCGA training set; and (e) KM survival curve distribution of 6-gene signature in the TCGA training set.

**Figure 4:** The construction of the nomogram. (a) Clinical features and the nomogram constructed by risk score; (b) correction chart of survival rate of the Nomogram; and (c) DCA curve.

**Figure 5:** Gene expressions of six CNV-related prognostic genes in RNA-seq. Some expression of the prognostic genes showed increased pattern in tumor tissues (CNV group). Compare with samples in Non-CNV group, expression in HMMR, GOLM1, and POSTN in tumor tissues (CNV group) were detected increases. *p*: *p* value using single-tailed *t*- test for paired data.

RETRACTED

**Figure 6:** Risk score distribution based on six prognostic genes in clinical validation cohort. (a) Comparison of risk scores between cancer and adjacent tissues. (b) ROC analysis of the six CRDS genes in the cancer and adjacent tissues. (c) Comparison of risk scores between cancer and adjacent tissues in different groups. (d) ROC analysis of the six prognostic genes in CNV group and Non-CNV group. *p*: *p* value using single-tailed *t*-test for paired data.

**Table 1:** Clinical sample information for three datasets.

Clinical features	TCGA-LUAD	GSE31210	GSE30219
PFS			
0	294	162	56
1	206	64	27
T stage			
T1	167		
T2	267		
T3	45		
T4	18		
TX	3		
N stage			
N0	324		
N1	94		
N2	69		
N3	2		
NX	11		
M stage			
M0	332		
M1	24		
MX	144		
Stage			
I	268		
II	119		
III	80		
IV	25		
X	8		
Gender			
Male	230		
Female	270		
Chemotherapy			
YES	175		
NO	325		
Radiation_therapy			
YES	58		
NO	361		
Unknown	81		
Age			
≤65	237		
>65	253		
Unknown	10		
Smoking∗			
1	71		
2	119		
3	129		
4	163		
5	4		
7	14		

∗Lifelong nonsmoker (less than 100 cigarettes smoked in lifetime) = 1; current smoker (includes daily smokers and nondaily smokers or occasional smokers) = 2; current reformed smoker for >15 years (greater than 15 years) = 3; current reformed smoker for ≤15 years (less than or equal to 15 years) = 4; current reformed smoker, duration not specified = 5; smoking History not documented = 7.

**Table 2:** Comparison of TCGA training set and validation set sample information.

Clinical features	TCGA-train	TCGA-test	*P*
PFS			
0	210	84	0.4632
1	140	66	
T stage			
T1	106	61	0.001
T2	199	68	
T3	36	9	
T4	9	9	
TX	0	3	
N stage			
N0	224	100	0.9006
N1	69	25	
N2	48	21	
N3	1	1	
NX	8	3	
M stage			
M0	242	90	0.1104
M1	14	10	
MX	94	50	
Stage			
I	187	81	0.1149
II	92	27	
III	53	27	
IV	14	11	
X	4	4	
Gender			
Male	161	69	1
Female	189	81	
Chemotherapy			
YES	118	57	0.4131
NO	232	93	
Radiation_therapy			
YES	41	17	0.9876
NO	252	109	
Unknown	57	24	
Age			
≤65	156	81	0.1485
>65	187	66	
Unknown	7	3	

**Table 3:** Clinical information of 20 LUAD patients.

No. of patients	Samples	Classification	Age	Gender	T stage	N stage	M stage	Tumor stage	Smoking	Family history
P2-41-13	P2-41-13-H3	Tumor	57	Male	1c	2	1a	IVa	Yes	No
P2-41-13	P2-41-13-H6	Adjacent normal	57	Male						
P2-41-13	P2-41-13-K1	Tumor	55	Male	1	0	0	I	Yes	No
P2-41-13	P2-41-13-K4	Adjacent normal	55	Male						
P2-41-14	P2-41-14-A1	Tumor	61	Female	1c	0	0	Ia3	No	No
P2-41-14	P2-41-14-A4	Adjacent normal	61	Female						
P2-41-14	P2-41-14-J9	Tumor	41	Female	2b	2	0	IIIa	No	No
P2-41-14	P2-41-14-K2	Adjacent normal	41	Female						
P2-41-31	P2-41-31-A1	Tumor	57	Male	1c	0	0	Ia3	Yes	No
P2-41-31	P2-41-31-A4	Adjacent normal	57	Male						
P2-41-31	P2-41-31-B10	Tumor	69	Female	2a	0	0	IB	No	No
P2-41-31	P2-41-31-C3	Adjacent normal	69	Female						
P2-41-31	P2-41-31-F3	Tumor	61	Female	1b	0	0	Ia2	Yes	No
P2-41-31	P2-41-31-F6	Adjacent normal	61	Female						
P2-41-31	P2-41-31-G2	Tumor	55	Male	2a	0	0	IB	Yes	No
P2-41-31	P2-41-31-G5	Adjacent normal	55	Male						
P2-41-32	P2-41-32-A10	Tumor	36	Female	Tis	0	0		No	No
P2-41-32	P2-41-32-B2	Adjacent normal	36	Female						
P2-41-32	P2-41-32-H8	Tumor	32	Female	Breast cancer lung metastasis					
P2-41-32	P2-41-32-J1	Adjacent normal	32	Female						
P2-41-32	P2-41-32-J2	Tumor	64	Female	1c	0	0	Ia3	No	No
P2-41-32	P2-41-32-J5	Adjacent normal	64	Female						
P2-41-32	P2-41-32-K1	Tumor	72	Female	1b	0	0	Ia2	No	No
P2-41-32	P2-41-32-K4	Adjacent normal	72	Female						
P2-41-33	P2-41-33-B9	Tumor	76	Male	1b	2	0	IIIa	Yes	No
P2-41-33	P2-41-33-C2	Adjacent normal	76	Male						
P2-41-33	P2-41-33-C8	Tumor	51	Male	2a	1	0	IIB	No	No
P2-41-33	P2-41-33-D1	Adjacent normal	51	Male						
P2-41-33	P2-41-33-D10	Adjacent normal	60	Female						
P2-41-33	P2-41-33-D7	Tumor	60	Female	1c	0	0	Ia3	No	No
P2-42-31	P2-42-31-D8	Tumor	55	Male	1	0	0	I	Yes	No
P2-42-31	P2-42-31-E1	Adjacent normal	55	Male						
P2-42-31	P2-42-31-E10	Adjacent normal	63	Male						
P2-42-31	P2-42-31-E7	Tumor	63	Male	1b	0	0	Ia2	Yes	No
P2-42-31	P2-42-31-H6	Tumor	56	Male	2a	0	0	IB	Yes	No
P2-42-31	P2-42-31-H7	Adjacent normal	56	Male						
P2-42-31	P2-42-31-K4	Tumor	53	Female	1b	2	0	IIIa	Yes	No
P2-42-31	P2-42-31-K5	Adjacent normal	53	Female						
P2-42-32	P2-42-32-A3	Tumor	74	Female	2a	0	0	IB	No	No
P2-42-32	P2-42-32-A6	Adjacent normal	74	Female						

RETRACTED

## Data Availability

The transcriptome sequencing data was uploaded to the Gene Express Omnibus (GEO) database under the accession GSE197346. To review GEO accession GSE197346, go to https://www.ncbi.nlm.nih.gov/geo/query/acc.cgi?acc=GSE197346. Enter token cbmvowqorlclfcj into the box.

## Supplementary Materials

Supplementary 1 Figure S1: Robustness of the prognostic model. A: Risk score, survival time and survival status and expression of 6-gene signature in the TCGA test set. B: ROC curve and AUC of 6-gene signature classification; C: KM survival curve distribution of 6-gene signature in TCGA test set. D: Risk score, survival time and survival status and expression of 6-gene signature in all TCGA data. E: ROC curve and AUC of 6-gene signature classification. F: KM survival curve distribution of 6-gene signature in all TCGA data sets.

Supplementary 2 Figure S2: Robustness of the prognostic model. A: Risk score, survival time and survival state and gene expression of 6-gene signature in the independent verification data set GSE31210. B: ROC curve and AUC of 6-gene signature in the independent verification data set GSE31210. C: KM survival curve distribution of 6-gene signature in the independent verification data set GSE31210. D: Risk score, survival time and survival state and 8-gene expression in the independent verification data set GSE30219. E: ROC curve and AUC of 6-gene signature in the independent verification data set GSE30219. F: KM survival curve distribution of 6-gene signature in the independent verification data set GSE30219.

RETRACTED

Supplementary 3 Figure S3: Comparison of clinical features. Comparison of the distribution of different clinical characteristics between two molecular subtypes in the TCGA dataset.

Supplementary 4 Figure S4: Comparison of molecular mutations. A: Distribution of different molecular mutations in high-risk groups in the TCGA dataset. B: The distribution of different molecular mutations in the low-risk group in the TCGA dataset. C: Comparison of high and low risk grouping immune scores in the TCGA data set. p: *p*-value derived from single-tailed t-test for paired data.

Supplementary 5 Figure S5: The presentation of risk score on clinical features in the TCGA dataset.

Supplementary 6 Figure S6: The distribution of risk score in clinical features and molecular subtypes of TCGA data.

Supplementary 7 Figure S7: Independence of risk models. A: Univariate survival Cox analysis of Clinical features and risk score; B: Multivariate survival Cox analysis of Clinical features and risk score.

Supplementary 8 Figure S8: Comparison of six genes expression in tumor tissues between CNV-group and Non-CNV group. A: In tumor tissues. B: in adjacent normal tissues.

Supplementary 9 Table S1: The gene expressions and CNV status of the six genes in TCGA datasets.

Supplementary 10 Table S2: The gene expressions and CNV status of the six-gene in 20 LUAD patients.
